The article "LINC00636 promotes lymph node metastasis and cervical cancer through targeting NM23" was retracted in 2024. Reasons: compromised peer review; no approval from an author; concerns about the authorship.

# LINC00636 promotes lymph node metastasis and cervical cancer through targeting NM23

**DOI:** 10.1042/BSR20200367

**Published:** 2020-10-30

**Authors:** Yue Zhong, Qiang Lu, Wei Qiu, Yan Luo

**Affiliations:** 1 Department of Ultrasound, Neijiang First People’s Hospital, Neijiang city, Sichuan Province, 641000, China; 2 Department of Ultrasound, West China Hospital of Sichuan University, Chengdu City, Sichuan Province, 610041, China

**Keywords:** cervical cancer, LINC00636, metastasis, NM23

## Abstract

**Background:** Metastasis is a major obstacle in treatment of cervical cancer, and long non-coding RNA (lncRNA) mediated regulatory effect on associated genes expression is found to be involved in metastasis. However, its mechanisms have not been fully elucidated.

**Materials and methods:** Specimens from patients with cervical cancer metastasis and non-metastasis were used to screen out candidate non-coding RNAs (ncRNAs) and possible downstream targets. And then, effects were determined *in vitro* and *in vivo* through knockdown and overexpression techniques.

**Results:** LINC00636 was significantly higher in serum and solid tumor cells of metastatic cervical cancer patients than non-metastatic patients. And knockdown of LINC00636 significantly suppressed invasion, proliferation of cervical cancer cells. NM23 expression was negatively regulated by LINC00636 and it mediated anti-tumor effects was partially blocked by overexpression of LINC00636.

**Conclusion:** LINC00636 might promote metastasis of cervical cancer cells through inhibiting NM23 expression.

## Introduction

Long intergenic non-coding RNAs (lncRNAs) are defined as autonomously transcribed non-coding RNAs (ncRNAs) longer than 200 nucleotides that do not overlap annotated coding genes.Long ncRNAs (lncRNAs) function broadly to tune gene expression by directly affecting nuclear architecture and by sequestering intracellular molecules or promoting their function, as well as more indirectly via the effects of their transcription or translation [1].

Cervical cancer is the third most common cancer and the second leading cause of cancer-related deaths in women worldwide [2,3]. Metastasis is one major challenge for cervical cancer treatment, as most cervical cancer-related mortality are caused by metastasis [4]. Unfortunately, there are currently no effective treatment options for preventing or inhibiting cervical cancer metastasis, in part because the mechanisms that underlie cervical cancer metastasis are not fully defined.

Previous investigations reported that several lncRNAs had been found to play a role in the metastasis of a variety of tumors. In the present study, a new lincRNA was found to be involved in the regulation of cervical cancer cells metastasis and its possible mechanism was initially explored.

## Materials and methods

### Human specimens

Specimens were obtained from three pairs of cervical cancer patients with or without metastasis confirmed by biopsy or surgery from 59 cervical cancer patients at Neijiang First People’s Hospital (see details in Table 1). This research has been carried out in accordance with the World Medical Association Declaration of Helsinki, and that all subjects provided informed consent. The present study has been carried out in accordance with the World Medical Association Declaration of Helsinki and was approved by the Ethics Committee of the Neijiang First People’s Hospital (Approval No. 2018-36).

**Table 1:** Characteristics of cervical cancer patients (*n*=59)

Characteristics	Variables	*n* (%)
Age (years)	Range, (means ± SD)	39–87 (56 ± 5.6)
Family history of cancer	No	46 (77.9)
	Yes	13 (22.1)
HPV	Positive	42 (71.2)
	Negative	17 (28.8)
TNM stage	I	20 (33.9)
	II	24 (40.7)
	III	9 (15.3)
	IV	6 (10.1)
Differentiation grade	Moderate	31 (52.5)
	Poor	28 (47.5)
Lymph node metastasis	Yes	15 (25.4)
	No	44 (74.6)

### Extraction of total RNA

Fresh tissue was collected, flash frozen and stored at −80°C. Hippocampi were dissected out in sterile saline after thawing the brains. Total RNAs of mice hippocampi were extracted by using TRIzol reagent (Invitrogen Life Technologies, U.S.A.) following the manufacturer’s protocol. The concentration and purity of the RNAs were checked by Nanodrop 2000 (Thermo Fisher Scientific, U.S.A.). For RNA sequencing, the RNA integrity was assessed by analyzing standard denaturing agarose gel electrophoresis and Agilent 2100 was used to determine RNA integrity number (RIN) value.

### Library construction, RNA sequencing and data analysis

First, rRNAs in samples from control and PM2.5 groups were removed. Then, the libraries for next-generation sequencing were prepared using the TruSeq RNA Sample Prep Kit (Illumina, U.S.A.) according to the manufacturer’s instructions. After enrichment and purification, the libraries were processed for sequencing by Shanghai Origingene Bio-pharm Technology Co. Ltd (Shanghai, China) according to available protocols. After quality control of the original data, the high-quality sequencing data are compared with the designated reference genome. The expression values were calculated by the StringTie tool, and tDESeq algorithm was applied to filter the differentially expressed genes.

### Cell culture

Hela, Caski, C3AA, Hcerpeic and SiHa cells were obtained from American Type Culture Collection (ATCC, Manassas, VA, U.S.A.), and maintained in Dulbecco’s modified Eagle’s medium with 10% fetal bovine serum (HyClone, Logan, UT) at 37°C in an atmosphere containing 5% CO_2_. A total of 5 × 10^4^ SiHa cells each well were cultured in a six-well plate at 37°C overnight until ∼60% confluence. The cells were then transfected with a mixture of 2 μg plasmid carrying LINC00636 and 6 μl Effectene transfections reagent (Qiagen China Co., Ltd., Shanghai, China) in 1 ml of fresh serum-free DMEM. For small interfering RNA (siRNA) transfections, cells were plated and in a six-well plate at a density of 5 × 10^4^ cells/well and cultured overnight at 37°C. Subsequently, 2 µl gene-specific siRNAs (see details in Table 2) (100 µM) each well were transfected in the presence of Opti-MEM medium (cat. no. 51985034; Gibco; Thermo Fisher Scientific, Inc.) using X-tremeGENE siRNA transfection reagent (cat. no. 4476093001; Roche Applied Science, Penzberg, Germany), according to the manufacturer’s protocols.

**Table 2:** Details of siRNA targeting NM23

Name	Sequence	Location
siRNA-1	Sense: 5′-CAGUGAGCGCAOCUUCAUUtt-3′	312 bp
	Antisense: 5′-AAUGAAGGUGCGCUCACUGtt-3′	
	Target sequence: 5′-AACAGTGAGCGCACCTTCATT-3′	
siRNA-2	Sense: 5′- AGAGCGCAGAGAAGGAGAUtt-3′	674 bp
	Antisense: 5′- AUCUCCUUCUCUGCGCUCUtt-3′	
	Target sequence: 5′-AAAGAGCGCAGAGAAGGAGAT-3′	
siRNA-3	Sense: 5′-UCUGAGUGGACAGAAUGUAtt- 3	981 bp
	Antisense: 5′-UACAUUCUGUCCACUCAGAtt- 3	
	Target sequence: 5′-AATCTGAGTGGACAGAATGTA-3′	
siRNA-NC	Sense: 5′-GACUUCAUAAGGCGCAUGC-3′	
	Antisense: 5′-GCAUGCGCCUUAUGAAGUC-3′	

### Immunohistochemistry and immunofluorescence

Sections were observed using an upright phase contrast light microscope (Nikon Corporation, Tokyo, Japan) at magnifications of ×200. The tissue specimens were fixed with 10% neutral formalin at room temperature for 15 min, embedded in paraffin and 5-mm-thick sections were prepared. Paraffin wax-embedded tissue sections were dewaxed, rehydrated (incubated in 100, 95, 80 and 75% series gradient ethanol at room temperature for 3 min each and then in distilled water for 10 min) at room temperature and microwaved at 95°C for 30 min in sodium citrate buffer (0.01 M, pH 6.0) to repair antigen epitopes. The tissue sections were incubated at 37°C for 10 min with 3% H_2_O_2_ and blocked by 5% normal goat serum (cat. no. AR0009; Wuhan Boster Biological Technology, Ltd., Wuhan, China) at 37°C for 10 min in order to eliminate endogenous peroxidase activity. Following this, tissue sections were incubated with primary monoclonal antibodies. The immunohistochemistry (IHC) staining score was reviewed by an expert panel of pathologists. Antibodies against NM23, β-actin, Bcl-2, BAX, cleaved caspase 3 and secondary antibodies were purchased from Abcam (Cambridge, MA, U.S.A.).

### Western blot

Cells are transfected with plasmid or siRNA (NM23 siRNA information in Table 2). Cell lysates (40 μg) were separated by 10% SDS/PAGE and transferred to polyvinylidene difluoride membranes (Immobilon-P membranes; EMD Millipore, Billerica, MA, U.S.A.). Membranes were blocked with blocking buffer (5% non-fat milk and 0.1% Tween-20 in TBS) for 1 h at room temperature. Following incubation with appropriate primary antibodies overnight at 4°C, membranes were then incubated with horseradish peroxidase-conjugated secondary antibodies (1:5000; cat. no. A16096; Invitrogen; Thermo Fisher Scientific, Inc.) at room temperature for 1 h, and protein bands were detected using Electrochemiluminescence Plus Western Blotting Detection system (cat. no. RPN2133; GE Healthcare Life Sciences, Little Chalfont, U.K.) with a ChemiDoc XRS+ imaging system (Bio-Rad Laboratories, Inc.).

### Invasion assay

Cells were transfected with LINC00636 expression plasmid or siRNA targeting LINC00636 (Genechem Co., Shanghai, China) using Lipofectamine 3000 (Invitrogen, Carlsbad, CA, U.S.A.) according to manufacturer’s instructions. After 48 h post-transfection, cells were subjected to invasion assay. Briefly, 10000 cells in growth medium without serum were seeded in the upper wells of invasion chambers (BD Biosciences, San Jose, CA, U.S.A.). The lower wells contained the same medium with 10% fetal bovine serum. After 24 h of cell seeding, the cells that had invaded to the lower side of the chamber were fixed with 2.5% glutaraldehyde, stained with 0.1% Crystal Violet, and counted.

### Luciferase reporter assay

Plasmids and/or nucleotides were transfected into SiHa cells that transfected with firefly luciferase reporter construct, which contained E-cadherin promoter. The *Renilla* luciferase plasmid was co-transfected as a transfection control (Promega). Cell extracts were prepared 72 h after of transfection, and the luciferase activity was measured using the Dual-Luciferase reporter assay system (Promega) according to manufacturer’s instructions. The luciferase activity was normalized by the activity of *Renilla* luciferase.

### Animal experiments

All xenograft models were generated using GFP-expressing SiHa cells (SiHa-GFP) in 6-week-old female BALB/c nude mice. For lymph node metastatic model, the SiHa-GFP cells (1 × 10^6^/50 μl per mouse) transfected with non-target control siRNA, siLINC00636 and plasmids overexpressing LINC00636 were directly injected into the foot pad of mice [5]. Tumor metastasis was monitored for seven weeks by IVIS Spectrum *in vivo* Imaging System (PerkinElmer, Utah, U.S.A.) and MRI (7.0-T MRI, Bruker Biospec 70/20USR, Germany). All animal experiments were performed in Central Laboratory of Neijiang First People’s Hospital and the experimental procedures were approved by the Ethics Committee of Neijiang First People’s Hospital (Approval No. 2019-035). The SiHa cells were suspended in Matrigel (BD Biosciences; Becton, Dickinson and Company, Franklin Lakes, NJ, U.S.A.) and subcutaneously implanted into the left flank of nude mice. Following implantation, tumor volumes were measured every 7 days until the mice were killed by CO_2_ at day 49 (no anesthetics used in this experiments).

### Statistical analyses

The Pearson’s correlation coefficient in R language package corrplot was calculated to measure the linear correlation of the expression levels of lncRNA and target genes. All statistical analyses were performed using Prism 5.0 software (GraphPad). The independent sample *t* test was used for comparing groups for statistical differences and *P*-values less than 0.05 were considered statistically significant. The data are presented as the mean with the standard deviation (SD) of at least three independent experiments.

## Results

### LINC00636 was overexpressed in cervical cancer with metastasis

First, whether cervical patients with lymph node metastasis or without metastasis was confirmed by Doppler ultrasound (Supplementary Figure S1). Next, increased expression of LINC00636 was found to be significantly up-regulated in cancer tissues (Figure 1A) and the serum (Figure 1B) of cervical cancer patients with lymph node metastasis compared with non-metastatic patients, which was similar with results downloaded from The Cancer Genome Atlas (TCGA) (Figure 1C) and LINC00636 overexpression have poor prognosis in cervical cancer patients (Figure 1D). In order to further study the role and mechanism of LINC00636 in tumor metastasis by *in vitro* experiments, we tested the expression of LINC00636 in several commonly used cell lines (Figure 1E), among which SiHa cells and C3AA cells had relatively higher expression. And SiHa cells were chosen to perform the next experiments. To further clarify the mechanisms of LINC00636, RNA-sequence analysis was also performed in three pairs of cervical cancer patients with and without metastasis and 20 genes with the most significant difference were shown in Figure 1F.

**Figure 1:** Cervical cancer patients with lymph node metastasis have higher expression of LINC00636 Compared with cervical cancer without lymph node metastasis, LINC00636 was significantly up-regulated in solid cancer cells (**A**) and serum (**B**) (*n*=15). (**C**) The results of TCGA database also showed that the expression of LINC00636 in tumor cells with metastasis was significantly higher than that in patients without metastasis and (**D**) LINC00636 overexpression have poor prognosis for **cervical cancer patients** by Kaplan–Meier analysis. (**E**) Relative expression LINC00636 in various common tumor cell lines. (**F**) Twenty genes with the most significant difference were identified from three pairs of metastatic and non-metastatic cervical cancer patients by RNA-sequence analysis. Values were presented as means ± standard deviations of three independent experiments unless indicated. *: *P*<0.05, ***: *P*<0.001. Independent *t* test.

### LINC00636 promotes SiHa cells proliferation through anti-apoptotic effect

To further clarify the role and mechanism of LINC00636 in cervical cancer cells metastasis, SiHa cells with relatively high expression levels were recruited for *in vitro* overexpression and knockdown experiment (Figure 2A). Compared with the non-target control (NC) siRNA group, at 72 h post-transfection, cell viability was found to be significantly inhibited in the LINC00636 knockdown group, while overexpression of LINC00636 significantly enhanced cell viability (Figure 2B) and cell proliferation (Figure 2C). Subsequent scratch experiments showed that overexpression of LINC00636 significantly enhanced the migration of SiHa cells, but LINC00636 knockdown had no effect on it (Figure 2D). Since LINC00636 plays a role in regulating SiHa cells viability and proliferation, the effect of LINC00636 on tumor cells apoptosis was further investigated through flow cytometry. As shown in Figure 2E, down-regulation of LINC00636 significantly increased the apoptotic rate of tumor cells, while overexpression of LINC00636 reduced spontaneous apoptosis. Western blot also showed similar results, knockdown of LINC00636 significantly increased cleavage-Caspase 3 which might be achieved by down-regulation of Bcl-2 and up-regulation of BAX, while LINC00636 overexpression showed the opposite effect (Figure 2F).

**Figure 2:** LINC00636 enhanced SiHa cells proliferation and immigration (**A**) Confirmation of knockdown and overexpression of LINC00636. Effect of LINC00636 on cells viability (**B,C**), migration (**D**) and apoptosis (**E,F**). Values were presented as means ± SDs of three independent experiments unless indicated. *: *P*<0.05, **: *P*<0.01, ***: *P*<0.001. Independent *t* test.

### Knockdown of LINC00636 inhibits cervical cancer cells lymphatic metastasis *in vivo*

In the present study, BALB/c nude mice were injected with SiHa-GFP cells without any treatment, LINC00636-deficient SiHa-GFP cells by siRNA and LINC00636 overexpressed SiHa-GFP cells, in order for nude mice to be subcutaneously tumorigenic, and observed at the same time. As depicted in Figure 3A, LINC00636-deficient cancer cells growth was significantly reduced and LINC00636 overexpressed cells growth was significantly enhanced, compared with the control. At day 49 post cells injection, the weight of the tumor in the LINC00636 knockdown group was also reduced compared with the control groups (Figure 3B). More importantly, the number of lymph node metastases was also significantly lower in the LINC00636 knockdown group than in the control group. However, the overexpression LINC00636 group did not significantly increase the number of metastases (*P*=0.0641) (Figure 3C). Expression of KI67 in various groups of cancer cells showed the similar results (Figure 3D). Lymphatic metastasis was confirmed by observation of SiHa-GFP cells in lymph node (Figure 3E).

**Figure 3:** LINC00636 knockdown inhibits SiHa cells growth and metastasis *in vivo* Tumor volume (**A**) and weight (**B**) were significantly lower in LINC00636 knockdown than control group. LINC00636 deficient cancer cells had fewer lymph node metastases (**C**) and lower KI67 expression (**D**) than control group. Lymphatic metastasis confirmed by observation of GFP (**E**). Values were presented as means ± SDs of tumor parameters from eight mice each group. **: *P*<0.01, ***: *P*<0.001. Independent *t* test.

### The inhibitory effect of LINC00636 on cervical cancer cells was achieved by suppressing expression of NM23

The above results showed that LINC00636 could promote cervical cancer cell proliferation and migration, which could be inhibited by knocking down LINC00636. Furthermore, the present study analyzed the correlation of differential genes expression that might be involved in cervical cancer cells metastasis shown in Figure 1 to find downstream targets of LINC00636. As shown in Figure 4A, the expression of LINC00636 and NM23 was significantly negatively correlated, which was further confirmed at transcription (Figure 4B) and translation level (Figure 4C,D). Compared with the control group, knocking down LINC00636 significantly increased the expression of NM23, while overexpressing LINC00636 suppressed its expression. Quantitative analysis also showed a significant negative correlation between both expression (Figure 4E). Next, luciferase reporter plasmids were constructed to assess whether LINC00636 has a direct regulatory effect on the promoter of NM23. Based on theoretically predicted binding site, a mutant NM23 promoter reporter vector was also constructed (Figure 4F). As shown in Figure 4G, overexpression of LINC00636 significantly inhibited the expression of wildtype (WT) NM23, but had no effect on mutant (MT), which proved that LINC00636 directly regulates NM23 expression through binding its promoter.

**Figure 4:** NM23 expression was regulated by LINC00636 (**A**) Correlation analysis between NM23 and LINC00636 by corrplot package in R. NM23 expression was suppressed by overexpression of LINC00636 and up-regulated by LINC00636 knockdown at mRNA (**B**) and protein level (**C,D**). (**E**) Pearson’s correlation analysis between mRNA level of NM23 and LINC00636 (*n*=59). (**F**) Predicted targeting site at promoter of NM23 by LINC00636 and its mutant design. (**G**) Luciferase reporter assay using LINC00636 overexpressing vector with WT and MT NM23 promoter reporter vector in SiHa cells. Values were presented as means ± standard deviations of three independent experiments unless indicated. ***P<0.001.

To further verify whether the inhibitory effect of LINC00636 on cervical cancer cells was achieved by regulating the expression of NM23, we further observed the effects of knockdown and overexpression of NM23 on tumor cells, and whether this effect was regulated by LINC00636. As shown in Figure 5A, knocking down NM23 could significantly inhibit the spontaneous apoptosis of cervical cancer cells, otherwise, overexpression of NM23 can significantly promote its apoptosis, which can be partially blocked by simultaneous overexpression of LINC00636. Cell proliferation (Figure 5B) and migration ability (Figure 5C) experiments also showed similar results. Further investigation found that NM23 may promote apoptosis (Figure 5D) of cervical cancer cells to down-regulate the cell viability (Figure 5E) through down-regulation of Bcl2 expression and up-regulation of BAX, while overexpression of LINC00636 can down-regulate NM23. The down-regulating effect of LINC00636 on NM23 expression was also confirmed in *in vivo* experiments (Figure 5F).

**Figure 5:** Impact of NM23 on cervical cancer cells can be partially blocked by LINC00636 NM23 deficiency could significantly attenuate SiHa cells apoptosis (**A**), promote cells invasion (**B,C**) and growth (**D**) and, while overexpression of NM23 had the opposite effect which could be partially blocked by overexpression of LINC00636. Western blot showed that impact of NM23 and LINC00636 SiHa cells might be through regulating Bcl2 and BAX expression (**E**). The *in vivo* xenograft showed that LINC006363 knockdown significantly up-regulated NM23 expression, while LINC00636 down-regulated it (**F**). Graphic summary of the present study, the LINC00636 plays a negative regulatory role in cervical cancer metastasis, which could be achieved by targeting NM23 (**G**). Values were presented as means ± SDs of three independent experiments unless indicated. *: *P*<0.05, **: *P*<0.01, ***: *P*<0.001.

## Discussion

Metastasis is the main cause of the low curative rate of oncologic tumors. Angiogenesis and lymphangiogenesis are early events in tumor metastasis, and the therapeutic effects of angiogenesis are limited by the close relationship between the vascular system and lymphatic system. Cervical cancer is a complex illness, many elements are involved in its occurrence. Several investigators have proposed that lncRNAs can be utilized for diagnosing and prediction of prognostication tumor [6]. Protein-coding genes have the responsibility of producing just 2% of the human transcriptions. However, the bulk of transcripts are ncRNAs encompassing microRNAs (miRNAs) and lncRNAs [6]. NcRNAs are protected and have clearly defined roles [7]. miRNAs are a category of small ncRNAs consisting of 19–23 nucleotides in length and substantially studied type of ncRNAs. LncRNAs are RNAs with 200 nucleotides (nt) in length, which are often transcribed by RNA polymerase II, having abundant structural characteristics of the mRNAs, consisting of a poly (A) tail, a 5′-cap and a promoter structure, and are in need of the conservative open reading domain [8]. To date, an overwhelming majority of lncRNAs have not been well-characterized. However, lncRNAs have been displayed to be drawn into almost every facet of gene regulation, containing epigenetic regulation, imprinting, trafficking of nucleus and cytoplasm, transcription, mRNA splicing [9–11]. Thus, lncRNAs were involved in many diverse biological processes, containing cell cycle, cell proliferation, apoptosis, differentiation etc [12–14].

It is common knowledge that invasion and metastasis were a root in poor clinical outcome and high relapse rate of cancer patients [15], which part related to some characteristics of cancer cells. It is well-known that recurrence and metastasis are the maximal obstacles to the therapy of cervical cancer. Therefore, hunting for the available markers of cervical cancer is essential for improving the prognosis. Several lncRNAs, including lncRNA-CRNDE [16], lncRNA-EBIC [17], lncRNA PCAT-1 [18], MALAT1 [19,20], GAS5 [21] and HOTAIR [22–24], have been found to be involved in cervical cancer metastasis and invasion through various mechanisms. In the present study, LINC00636 was found for the first time in the blood of patients with cervical cancer associated with lymph node metastasis and in tumor cells. SiHa cells with overexpressed and deficient LINC00636 were used to investigate its impact on cervical cancer cells proliferation, apoptosis, migration and invasion, it was found that LINC00636 might promote cervical cancer cell growth and metastasis by inhibiting apoptosis of cervical cancer cells. These results suggest that the increased expression of LINC00636 is predictive of the poor prognosis for cervical cancer patients. At the same time, LINC00636 can be used as an indicator of prognosis and a new intervention target for cervical cancer. However, the mechanisms of LINC00636 elevation in patients with metastatic cervical cancer needs further study. Previous studies found that LINC00636 is up-regulated in human epidermal growth factor receptor-2 (HER-2) highly expressed breast cancer subtype [25] and pancreatic ductal adenocarcinoma [26] and could be the indicator of prognosis, which are consistent with results in this study.

Since lncRNAs usually function by regulating the expression of downstream genes, we next screened its possible targets by analyzing the correlation between lncRNAs and the expression of key molecules of signaling pathways involved in cervical cancer metastasis. NM23 was initially found in metastatic cell lines by Steeg et al. in 1988 and was the first of what has become a field of over 20 known metastasis suppressor genes [27,28]. In humans, there are ten genes belonging to the *NM23* gene family, of which the two most abundantly expressed are NM23-H1 and NM23-H2 that encode the A and B subunits of nucleoside diphosphate kinase, respectively [29]. As a recognized cancer suppressor gene, NM23 expression has been proved to be negatively correlated with metastasis of various cancer including gastric cancer [30] and cervical cancer [31]. However, its regulation has not been fully understood. The present study found that overexpression of LINC00636 could down-regulate NM23 expression through binding it, and then, NM23 mediated anti-tumor effect was thus weakened.

In summary, the present study found for the first time that LINC00636 plays a negative regulatory role in cervical cancer metastasis, which may be achieved by binding to NM23 genomic DNA and inhibiting its expression (Figure 5G).

## Supplementary Material

Supplementary Figure S1

## Data Availability

All data generated or analyzed during the present study are included in this published article.

## Abbreviations

BAX: BCL2-Associated X
Bcl-2: B-cell lymphoma-2
lncRNA: long non-coding RNA
miRNA: microRNA
ncRNA: non-coding RNA
siRNA: small interfering RNA
